The article "Apoptosis Activation and Autophagy Inhibition of Chondrocytes by Leptin by the Upregulation of LOXL3 in Osteoarthritis Pathogenesis" was published in 2022. Journal: J Healthc Eng.

# Apoptosis Activation and Autophagy Inhibition of Chondrocytes by Leptin by the Upregulation of LOXL3 in Osteoarthritis Pathogenesis

**DOI:** 10.1155/2022/4026128

**Published:** 2022-01-07

**Authors:** Qianhao Wei

**Affiliations:** Central South University Staff Hospital, Changsha, China

## Abstract

**Background:**

Osteoarthritis is one of the usual chronic musculoskeletal dysfunctions. It is one of the primary leading causes which leads to limitation of movement and absenteeism in the working adult population. Chondrocytes are the singlecellular-based component found in the cartilage which has an important role in the degradation of the cartilage. In recent studies, autophagy is observed to protect the human chondrocytes from stress.Leptin an adipokine managing food consumption and energy outlay. Chondrocytes indicate prolonged isoform of the leptin receptor where inside these cells theleptin signals individually or combine with the remaining molecules and promptthe indication of the pro-inflammatory molecules and cartilage disintegration enzymes.

**Materials and Methods:**

mRNA expressions of Lysyl oxidase-like 3 in tissues of cartilage and concentration of leptin from synovial fluidwere measured from all samples from disease-induced groups, sham group, and RAPA-treated groups via RT-PCR and immunoassays. Histopathological analysis was also performed post-induction of the rat osteoarthritis model by the anterior cruciate ligament transection method. Western blot analysis was done, and expressions were analyzed by autophagy and apoptosis regulatory markers. Cell apoptosis and cell survival were evaluated with the help of flow cytometry, respectively, in all groups.

**Result:**

mRNA of LOXL3 was increased in osteoarthritis models which were directly related to leptin concentration in SF. ACLT surgery caused an increase in cleaved caspase 3 protein levels, while a significant reduction in Bcl-2, Beclin1, and LC3 I was noted (figure 4,5). When LOXL3 was silenced in the ACLT group and leptin-treated group apoptosis was inhibited and autophagy, cell proliferation was promoted in primary chondrocytes. A significant increase in LOXL3 caused inhibition of autophagy in chondrocytes.

**Conclusion:**

LOXL3 has stimulated apoptosis while inhibited autophagy in chondrocytes; hence LOXL3 is a prominent target for treating osteoarthritis. Keywords:chondrocytes, LOXL3, Leptin, osteoarthritis, qRT-PCR, ACLT, mRNA.

## 1. Introduction

The persistent ailment of osteoarthritis comprises of cartilage, subchondral bone, and synovium. Osteoarthritis shows the primary indication of swelling of joints along with pain and the deformities and frigidness along with dysfunction. Such disorders are usual among the elderly population where the maximum occurrence of it is seen, and the disabilities can be found more in women as compared to men. The osteoarthritis critically affects the physical as well as the mental health of the patients [1]. Osteoarthritis is one of the usual occurrences which is a chronic musculoskeletal dysfunction. Epidemiological research predicts approximately 43 million patients are found in the United States which is 15% of the global population [2, 3]. This is a principal source of restricting the activity and makes the working adults suffer from absenteeism which is connected with a notable reduction in the purpose among the older population. The collapse of chondrocytes to preserve between the synthesis as well as decay of extracellular matrix elements results in osteoarthritis [4]. There is a minute increment in the enzymatic role caused by the trauma associated with the microfracture or the inflammation, which also permits the development of the damaged particles that can be immersed by the inhabitant macrophages [5].

The article "Apoptosis Activation and Autophagy Inhibition of Chondrocytes by Leptin by the Upregulation of LOXL3 in Osteoarthritis Pathogenesis" was published in 2022. Journal: J Healthc Eng.

In the previous research, it has been proposed that the pathogenesis of osteoarthritis is connected with the deformation of joints which occurs because of the vitiated cartilage. Although, multiple studies with deep research also demonstrate the crucial character of inflammatory reaction in the pathogenesis of osteoarthritis [6, 7]. TNF-*α* is the main inflammatory element of cartilage deformation in osteoarthritis. The researches demonstrate that TNF-α is dispersed at multiple levels inthe articular cartilage subchondral bone and synovium. It encourages the unfettering of fibroblast adhesion molecules and secures to operate the vascular endothelial cell sticking molecules to concentrate the white blood cells in the articular space [8]. Chondrocytes are majorly responsible for the synthesis and the variation of the extracellular matrix through the autophagy and apoptosis [9]. Leptin has been examined as an adipokine with its pleiotropic effects since it was instituted in the year 1994. The leptin signaling system is dependent on the communication with the leptin receptor which is LEPR. The hindrance of leptin signaling has defensive effects on these disorders demonstrating the major role of leptin in the decay of cartilage [10].

The human lysyl oxidase-like 3 (LOXL3) gene was primarily recognized by the EST database probe. At initial level, the activity of LOXL3 as the amino oxidase was established on the homology with different members of the class. Lately, additional researches related to LOXL3 review the formation, role, as well as action and its development along with different pathologies [11]. LOXL3 can be transported to the nucleus because of the bipartite nuclear localization sign (residues 293-311), which consists of a couple of basic amino acid clusters [12]. Moreover, there is an assumption of nuclear transmitting signal in the N-terminal area which partly coincides with the signal peptide [13].

The article "Apoptosis Activation and Autophagy Inhibition of Chondrocytes by Leptin by the Upregulation of LOXL3 in Osteoarthritis Pathogenesis" was published in 2022. Journal: J Healthc Eng.

It has been reported that LOXL3 is related to a wide variety of disorders found in both animals and humans. LOXL3 can be found in snails where it lowers the rate of E-cadherin in the development of cancer [14], to produce the autophagy of chondrocytes in osteoarthritis [15] and to perform a crucial role during the control of integrin signal process for accurate position and anchoring of myofibers [16]. The appearance of LOXL3 was observed to be remarkably diminished at both mRNA and the levels of protein in the vaginal tissues found in the patients with the pelvic organ displacement.

## 2. Materials and Methods

### 2.1. Experimental Design

Rats weighing 200 g were collected from the company. These rats were induced with experimental osteoarthritis via anterior cruciate ligament transection. 6 rats were divided in each group randomly with a total being 18 rats collectively in 3 groups: control group (sham-operated), RAPA (ACLT+rapamycin) group, and ACLT+vehicle group. Post-anesthesia, the right knees of rats were shaved, and 70% ethanol was applied as a disinfectant. In the sham group, the joint was opened via a partial dislocation of the patella; then the wound was closed. In other groups, ACLT was performed as mentioned by Stoop R et al, 2001 [17]. Rats in the RAPA and ACLT + vehicle group received 0.3 ml DMSO vehicle (0.4% in PBS) and 1 mg/kg body weight rapamycin as an intraperitoneal injection. Post 10 weeks of the surgery, the rats were euthanized.

SF (synovial lavage) fluid was obtained from rats; cells were isolated post centrifugation. The knee joint cavity was washed two times by aspirating the space with 100 mL of PBS having 4 mM EDTA (ethylenediaminetetraacetic acid). Then the skin over the knee was removed and the knee ligament was dissected. Collected synovial lavage fluid was combined and stored at −20°C for future analysis. The procedures of experimentation on animals were approved by the animal ethical committee. 

### 2.2. RNA Isolation

Total RNA was collected with help of TRIzol reagent (Fischer Scientific) from tissues and cells with help of cDNA kits following the manufacturer's instructions. qRT-PCR was performed using PCR instrumentation where GADPH is the internal control and the DDCt method was used for the estimation of gene expression.

### 2.3. Histological Analysis

Knee joints were obtained and then fixed in 4% PFA where decalcification was done for 2 weeks at 4 degrees. Post dehydration tissues were soaked in ethanol with gradual concentrations which were fixed with paraffin. 5 mm sections were cut and deparaffinized using Safranin-fast green.

The article "Apoptosis Activation and Autophagy Inhibition of Chondrocytes by Leptin by the Upregulation of LOXL3 in Osteoarthritis Pathogenesis" was published in 2022. Journal: J Healthc Eng.

### 2.4. Immunofluorescence

Tissue sections were exposed to anti-LOXL2-specific antibodies where primary antibodies were identified and combined with conjugated anti-biotin antibodies. DAPI was added to all samples along with an anti-fade reagent, and the sections were analyzed under a fluorescent microscope. Regions were identified for any signs of inflammation, apoptosis, degeneration, etc.

### 2.5. Production of Lentivirus

 LOXL3 gene of the rats was synthesized using Thermo Fischer Scientific and then cloned into lentiviral vector for construction of pLvx-AcGFP-C1/LOXL3. In the normal control group, pLvx-AcGFP-C1 was used for the generation of mock viruses.

### 2.6. Isolation of Chondrocytes

In the osteoarthritis model of rats, the tissues from cartilage were isolated and cut into small pieces of <1 mm. 0.4% collagenase solution was used for digestion of tissues for 5 hours at 37°C. After centrifugation, the cells were cultured in DMEM/F12 medium with antibiotics and 10% fetal bovine serum. Isolated chondrocytes were then seeded in 6-welled plates with rapamycin, lentivirus, and leptin (Thermo Fischer Scientific).

### 2.7. Analysis of Apoptosis and Cell Proliferation

Cells were stained twice, with Annexin V-FITC and propidium iodide, and the analysis was done via flow cytometry (Bio compare). The PI negative and Annexin V-FITC (positive) cells were counted as apoptotic cells. Analysis of cell proliferation was determined with the help of Cell Counting Kit-8 Assay kits at 24, 48, and 72 hours, respectively, post-leptin treatment. Post 1 hour, CCK-8 solution was added to the culture medium and incubated. The absorbance was then noted at 450 nm wavelength via a microplate reader. Wells were measured for treatment and all experiments were run thrice for accurate results.

### 2.8. Western Blotting

Preparation of cell lysate was done by RIPA buffer and cultured cells (pH 7.2, 50 mM Tris HCl, 1% sodium deoxycholic acid, 150 mM NaCl, 1% Nonidet P-40, and 0.05% SDS). The same amount of protein was used for SDS-PAGE which was transferred to a nitrocellulose membrane. The membranes were then probed with primary antibodies which corresponded to secondary antibodies (horseradish peroxidase-conjugated). Using the chemiluminescence system, blots were detected and enhanced. Anti-Bcl-2 and anti-LOXL3 were the primary antibodies from Bio-compare. The antibodies used against LC3 and caspase-3 were obtained from Sigma-Aldrich. AKT, p-p70S6K, GAPDH, p70S6K, and p-AKT (S473) were obtained from Thermo Fischer Scientific.

The article "Apoptosis Activation and Autophagy Inhibition of Chondrocytes by Leptin by the Upregulation of LOXL3 in Osteoarthritis Pathogenesis" was published in 2022. Journal: J Healthc Eng.

### 2.9. Statistical Analysis

The statistical analysis was performed using SPSS. The data presented are as ± 95% confidence interval. Differences in results between groups were determined via the one-way ANOVA test. *P* < 0.05 was statistically significant, and the relation between the two factors was determined via correlation analysis.

## 3. Result

### 3.1. Analysis of LOXL3 and Leptin via the Experimental Rat Model of Osteoarthritis

To explain the relation between leptin and LOXL3 in osteoarthritis, a rat model was established with ACLT. Rats were evenly divided into three groups; control group (sham operated), RAPA (ACLT + rapamycin) group, and ACLT + vehicle group. Histopathological assessment was performed ten weeks post-surgery with Safranin staining. A significant degeneration was noted in the ACLT + vehicle group showing a decrease in chondrocytes. RAPA injection has shown a significant reduction in osteoarthritis changes by decreasing severity. In joint and cartilage samples, leptin and LOXL3 mRNA concentration and synovial fluid lavage levels were measured. The leptin and LOXL3 mRNA levels were reduced in the ACLT group while attenuated in the RAPA group. A level of correlation was observed between the leptin and LOXL3 levels. The data have indicated that high LOXL3 and leptin levels were linked with changes like osteoarthritis (Figures 1–5).

### 3.2. LOXL3 Expression Induced by Leptin in Cultured Primary Chondrocyte

To explore leptin and LOXL3 functions in the arthritis model, the chondrocytes were primarily collected via sham-operation in the rat knee joint. Immunohistochemistry staining by SOX931 and II30 was done for the identification of isolated chondrocytes (Figure 6). The isolated chondrocytes from ACLT surgery in the knee joint were then treated with 5 ng/ml to 20 ng/ml leptin. It was noted that the level of LOXL3 protein in chondrocytes was higher than in the control (sham-operated) group. Exposure to leptin caused a significant increase in the LOXL3 expression according to dosage (Figure 7).

The primary chondrocytes were identified from the sham-operated group and stained with anti-Collagen II (Thermo Fischer) which is an indicator of chondrocytes.

### 3.3. Promotion of Proliferation and Apoptosis Inhibition in Chondrocytes by LOXL3 Silencing

To study the difference in biological behavior in chondrocytes due to LOXL3, the isolated chondrocytes from the ACLT surgery in the knee joint were treated with 20 ng/ml leptin and siNC/siLOXL3. Measurement of relative proliferation was done using the CCK-8 assay as shown in Figure 7 which also demonstrated an increase in the levels of proliferation in chondrocytes. When the chondrocytes were transfected with siNC and the control group, it was observed that therewere an increased level of apoptosis (as identified by cleaved capase-3) and suppressed levels of Bcl-2 protein noted. Contrary to the siLOXL3 transfected chondrocytes, the levels of proteins with an apoptosis marker were reduced significantly whereas the anti-apoptosis expressions were significantly increased. Hence, the data have shown inhibition of apoptosis due to the effect of siLOXL3 on chondrocytes (Figure 8).

The article "Apoptosis Activation and Autophagy Inhibition of Chondrocytes by Leptin by the Upregulation of LOXL3 in Osteoarthritis Pathogenesis" was published in 2022. Journal: J Healthc Eng.

## 4. Discussion

Many studies have reported an overexpression in leptin in the pathogenetic studies in the osteoarthritis model. The cell death of chondrocytes is a major step in osteoarthritis which induces both autophagy and apoptosis. A lot of evidence has implied that regulation of apoptosis and autophagy is due to leptin and various types of cells. Therefore, we have tried to explore the effects on apoptosis and autophagy in chondrocytes in the pathogenesis of osteoarthritis due to leptin.

Firstly, it was noted that during RT-PCR there is an overexpression of LOXL3 in osteoarthritis patients [18]. The presence of LOXL3 in human tissues has hinted about their role in craniofacial cartilage maturation but is highly expressed in the damaged cartilage of patients suffering from osteoarthritis. A strong relation was found between the mRNA level of LOXL3 and leptin SF in cartilage in samples from the rat model of osteoarthritis. For further investigating the relationship between leptin and LOXL3, isolated chondrocytes were treated with leptin doses. Here, the exposure of leptin has shown overexpression of LOXL3 as per dose dependency. The results have also suggested that LOXL3 plays a significant role in the pathogenesis of leptin-associated osteoarthritis. Apoptosis in chondrocyte is a prime factor involved in the pathogenesis of osteoarthritis. When primary culture was isolated from chondrocyte cells of the rat model (osteoarthritis), a significant reduction in apoptosis was noted in siLOXL3 treatment, and cleaved caspase-3 expression was also found reduced but a significant increase in Bcl-2 expression, as well as cell survival, was found.

More research is required for exploring the mechanisms involved in the process as it was noted that leptin might be a crucial factor in LOXL3 expression, thereby promoting apoptosis in chondrocytes. Some studies have quoted that autophagy might be a defense mechanism of chondrocytes for protecting the chondrocytes from stress and progression of osteoarthritis. Suppression in the expression (western blot) of Beclin-1 and LC3 is due to the damage caused by osteoarthritis (Figure 5). Thus, in this study, the high expression of LOX3 was noted suppressed cell autophagy in the osteoarthritis rat model (Figures 3 and 4). mTOR-dependent signaling due to LOXL3 might suppress the autophagy in chondrocytes. As leptin inhibited autophagy in T cells but induced autophagy in the heart, liver, and skeletal muscles [19]. Thus, it was found that leptin shows tissue-specific autophagy actions. 

The article "Apoptosis Activation and Autophagy Inhibition of Chondrocytes by Leptin by the Upregulation of LOXL3 in Osteoarthritis Pathogenesis" was published in 2022. Journal: J Healthc Eng.

## 5. Conclusions

We conclude that an increase in leptin in rats who were suffering from osteoarthritis have increased the LOXL3 expressions. This led to apoptosis in chondrocytes which might have triggered the mTOR pathway thereby inhibiting autophagy in chondrocytes. Hence LOXL3 is a probable therapeutic target for treating osteoarthritis. 

## Figures and Tables

**Figure 1:** Histopathological analysis of tissues from all groups.

**Figure 2:** LOXL3 mRNA levels in all groups after activity.

**Figure 3:** Leptin (ng/ml) levels.

**Figure 4:** Expressions of LOXL3, Bcl-2, cleaved caspase-3, and GADPH as measured by western blot.

**Figure 5:** Expressions LC31, Beclin-1, and GADPH as measured by western blot.

**Figure 6:** Cultured primary chondrocytes from the sham group after staining with anti-Collagen II.

**Figure 7:** Relative cell proliferation percentage.

**Figure 8:** Relative proliferation level for LOX, Bcl-2, and cleaved caspase-3 in all groups.

## Data Availability

The data used to support this study are available upon request to the author.
